# A Digital Way for Fabricating a Resin-Bonded Fixed Partial Denture Combined with Periodontal Splint in the Mandibular Anterior Region

**DOI:** 10.1155/2022/6254551

**Published:** 2022-08-28

**Authors:** Xiaorui Shi, Yalin Zhan, Feng Liu

**Affiliations:** ^1^First Clinical Division, Peking University School and Hospital of Stomatology, Beijing, 100081 Beijing, China; ^2^National Clinical Research Center for Oral Diseases, Beijing, 100081 Beijing, China; ^3^National Engineering Laboratory for Digital and Material Technology of Stomatology, Beijing, 100081 Beijing, China; ^4^Beijing Key Laboratory of Digital Stomatology, Beijing 100081, China

## Abstract

Teeth loosening are caused by insufficient supporting tissue, inflammation of periodontal tissue, or occlusal trauma, which is one of the main clinical symptoms of periodontitis. A digital technique for fabricating resin-bonded splinting fixed partial dentures (S-FPDs) is presented. It restores the missing mandible anterior teeth and splints the adjacent periodontally mobile teeth of the patient at the same time. The S-FPDs is designed and fabricated by computer-aided design and computer-aided manufacturing (CAD/CAM) technology with flexible PMMA material. The workflow is straightforward, convenient, and accurate. Meanwhile, the restoration can meet the esthetic requirements and help with the stability of adjacent loosening natural teeth spontaneously. It could be considered a medium-term provisional restorative treatment option, but further controlled investigations still be needed.

## 1. Introduction

Severe periodontitis was the sixth most prevalent disease worldwide, with a global prevalence of 11%. Periodontitis is mainly a chronic inflammation of the periodontal supporting tissue caused by local factors. It is caused by certain bacteria and by local factors progressing from gingivitis to periodontitis and leading to the morbidity and loss of the tooth [1].

Attachment loss is the result of destruction of the periodontal supporting tissue. As a result of the progressive loss of attachment tissue, the teeth involved in the disease process eventually exhibit increased tooth mobility. Thus, the reduction of mobility is an important objective of periodontal therapy. Root planning, curettage, oral hygiene, and surgery may cause teeth to tighten as inflammation is resolved. Occlusal adjustment, periodontal orthodontics, and restorative dentistry may alter occlusal relationships and redirect forces, thereby reducing traumatism, which in turns improve the tooth looseness.

Increasing the support of loose teeth may also increase their firmness; the device used for such treatment is the splint. Grant defined splint is any appliance that joins two or more teeth to provide support. The American Academy of Periodontology described splint as a rigid flexible appliance used to stabilize and protect an injured part [2]. Literature [3] indicates that the main reasons for periodontal splinting are primary and secondary occlusal trauma, and progressive mobility. It may also be used to maintain periodontally migrated teeth that have been repositioned. Therefore, splint is considered to be an accepted practice to treat mobile teeth, particularly lower incisors, to maintain the patient's natural dentition as long as possible. In conclusion, a periodontal splint is an appliance that treats and fixes loose teeth.

Splint should be esthetically acceptable and biologically compatible, not interfere with other treatment, simple, economic, stable, and efficient. From the patient point of view, splint should protect gingiva from food impaction, be rigid, durable, and should not impair phonetics. According to the duration of use, it can be classified into short-term temporary splint (worn for less than 6 months), medium-term provisional splint (worn for months to several years), and long-term permanent splint (maintain long-term stability). According to the type of material, it can be divided into external and internal splints. The splints commonly used, such as ligature wires, night guards, interim fixed prostheses, and composite resin restorative material with or without wire or fiber inserts, are of external type. Among the type mentioned above, fiber-reinforced composite periodontal splint (FRC) is one of the most popular splint in periodontal clinical treatment, but it is difficult to adapt to the contour of lingual surface and well-polished, so the patient reports less comfort. It also has ultra-high tensile strength and high elastic modulus, and has stable chemical properties and good biocompatibility.

Moreover, periodontitis is the leading cause of tooth loss in adults. Specifically, plaque can cause the gums to recede, and damage to the alveolar bone can cause teeth to become loose or fall out. When tooth loss happens in the lower anterior teeth region, patients are more inclined to choose fixed restoration or implant restoration considering comfort and aesthetics. However, when tooth loss is due to severe periodontitis, the periodontal support tissue of adjacent teeth is compromised [4], so there is a risk to be the abutment of fixed restoration. Moreover, due to the severe bone loss, bone augmentation will be required during implant surgery, as well as soft tissue transplantation. This will for sure increase the complexity of the treatment and postoperative reflection. In addition, the average width of mandibular incisors is around 5.5 mm [5], the space of which cannot meet the requirements for implant placement most of the time. Besides, there is common crowding in mandibular anterior region. The twisting of adjacent teeth will make the space even smaller, then strategic extraction of adjacent teeth is often required for implant placement. Thus, extraction and implant or removable partial denture therapy are not viable alternative treatment options, because of patient- and site-related factors.

In this case, clinicians have to combine partial fixed dental prostheses and periodontal splint together, acting as a medium-term provisional restorative treatment method. Extracted teeth and composite resin have been used for pontics allowing immediate esthetic recovery, while loose adjacent teeth have been reinforced with splinting. At the early time, the direct-bonded method of metal reinforcement with artificial acrylic teeth was reported. Then, clinicians started to use fiber-reinforced composite (FRC) most of the time [6, 7]. Reviewing literature [7], a combination of a FRC-bonded splint, bridge, fiber post, and/or resin veneer for minimally invasive prosthodontic treatment in the aesthetic zone is a good choice for periodontal patients. Others reported [8] the use of resin-bonded fixed partial dentures (RBFPDs) as a solution, with a 5-year survival rate from 84.41% to 91.4%.

Although it can provide healing of supporting structures, facilitate the stability, and improve the esthetic, there are still some disadvantages. Despite the requirement of good oral hygiene maintenance and carefully control of occlusion, if the restoration is made indirectly, conventional physical impression will be needed. For periodontally compromised dentitions, conventional impression might be inaccurate so the seating of the restoration would be problematic. According to literatures [9, 10], wide interdental undercuts resulting from attachment loss in periodontally compromised patients are a problem for impression taking with elastomers as the material flow into the undercuts and sets. Due to the high tear strength of impression materials (polyvinylsiloxane or polyether), the removal of the impression especially in cases with severe undercuts is difficult and may result in permanent distortion and tear outs. Considering the acquirements of the restoration, it is not an option to block out the undercuts, so some clinicians finish the treatment intraorally under rubber dam isolation. Since the restoration is made directly, it is difficult to achieve proper contour of the splint part at the gingival margin, especially in the interproximal areas. Meanwhile, longer time of chair-side manipulation is often acquired, as well as high technical sensitivity, which is difficult for unexperienced dentists and less comfort to the patient.

Digital procedure seems to be a better solution. It improves efficiency and reduces time. The application of 3D digital system can simplify the tedious 20 processes into one step, and the whole process can be completed in one hour. Obviously, incorporation of digitized technologies becomes the changing trend in dentistry, as well as in periodontology. On the one hand, dentists start with digitizing patient records, storing radiographs and clinical photographs for ease of storage and quick checking, then benefit for better patient management. Live videos, three-dimensional animations, voice-activated software, and virtual consultations will help to build better report with patients as well as educate and motivate them. 3D advancement periodontal probing, AI technology in detection of dental plaque, and T-Scan system can also help with the diagnosis.

On the other hand, laser, AI technology, 3D Bioprinting, and computer-assisted anesthetic delivery can utilize the treatment procedure, of which the most widely used is digital radiography and intraoral scanning. Digital radiography uses an X-ray-sensitive plate that captures data directly during patient exams and transmits it to a computer system without the use of an intermediate cassette. They can be very useful in assessing pathological abnormalities and restorative treatment of periodontally involved dentations.

Intraoral scanning is the basis of digital design and manufacture in dentistry. Intraoral scanners are the basis for the realization of oral digital diagnosis and treatment. Studies have confirmed both reliability and validity in use on single teeth and dentition [11]. Mangano et al. [12] postulated that optical impressions obtained from intraoral scanning can simplify the following treatment, especially for complex situations such as large undercuts. Moreover, it is clinically accurate in capturing the contour of gingiva near the teeth and palatal mucosa [13]. This technology can assess changes in the soft tissue around a single tooth or implant after mucogingival surgery and implantation [14]. Some researchers [15] even found that digital intraoral scanning is more accurate than using a periodontal probe to measure the keratinized tissue width.

Combined intraoral scanning with computer-aided design and computer-aided manufacturing (CAD/CAM) technology, some clinicians [16] induced a method to fabricate periodontal splint by titanium alloy materials without tooth loss. Although further controlled investigation should be needed, the patient who was treated by that method showed acceptable results on 6 months recall. But for the situation with tooth missing, the alloy material is obviously unable to meet the esthetic requirements. If combined application of other materials (such as resin or ceramic), bonding area might become the weak link, which affect the longevity of the restoration. Not to mention interdental loss of periodontal tissue would have an effect on the design, the alloy material would be visible if extended too far.

To sum up, for periodontally involved patients with lower anterior teeth missing combined with loosen adjacent teeth, this article describes a digital way for fabricating a resin-bonded fixed partial denture together with periodontal splint based on CAD/CAM technology from polymethylmethacrylate (PMMA), in order to restore the missing teeth and splint the mobile teeth at the same time. PMMA is a high molecular polymer with the advantages of high transparency, low price, and easy machining. This treatment could be considered a medium-term provisional restorative method for the patient when other treatment options, for example, implantation or removable partial denture, are rejected for various reasons.

## 2. Techniques

The technique is described for a 45-year-old female patient who had a chief complain of mobile mandibular anterior teeth as well as tooth missing (Figure 1(a)). She had irregular periodontal treatment in the past few years and lost her mandibular central incisor 6 months ago. Her remained mandibular incisors had moderate bone loss (Figure 1(b)) with 1-2 degree mobility and crowding (Figure 1(c)). 6 weeks after initial periodontal therapy, the infection was controlled but no change was found in mobility. The patient had an urged esthetic demand while preserving the existing teeth.

The resin-bonded splinting fixed partial dentures (S-FPDs in short) technique was used as follows:

1. Get the digital model

Perform intraoral scan (TRIOS; 3Shape A/S) to both dentitions and get the digital model as well as the maximum intercuspal position digital bite registration (Figure 2). The standard tessellation language (STL) file was imported into the CAD software (exoCAD; excad GmbH).

(2) Design the restoration

Design the S-FPDs in the CAD software. It ranges from canine to canine in the lingual side, with the minimal thickness of 1 mm and 4 mm height. The ranges might be altered according to the loosening situation. This patient only got mobility at lower anterior incisor. If there are too many mobile teeth to form a stable fixation, this method should not be considered. For CAD/CAM PMMA materials, no thickness requirements were found for fabricating periodontal splints. However, according to the data provided by the manufacturer, when used for provisional crown restoration, the minimum thickness of the axial wall recommended for this material is 1 mm. As a reference, it is taken as the minimum thickness of the designed S-FPDs restoration. The margins were designed without extending beyond the incisal edge and cingulum (Figure 3(a)). Missing anterior tooth was designed with a slight rotation according to space and esthetic. The restoration was seated lingually.

(3) Fabricate the restoration

The S-FPDs was fabricated from multilayered PMMA (Flexible PMMA 98x20, Adite), milled with 5-axis inlab milling unit (CEREC MC X5, Dentsply Sirona). Separate the sprue, adjust, finish, and polish the lingual and labial surface with PMMA series adjusting and polishing burs (PMMA Adjusting and Polishing Kit, Hager & Meisinger GmbH). Then, perform airborne-particle abrasion to the intaglio surface with aluminum oxide (50 *μ*m, 2 bar) and clean it with compressed air (Figure 3(b)).

(4) Cement the restoration

Apply a bonding primer on the intaglio surface of the restoration (SR Connect, Ivoclar Vivadent) and light cure. The lower anterior teeth were isolated by rubber dam. The enamel surfaces on the lingual side were subsequently etched with 35% orthophosphoric acid (Gluma Etch, Heraeus) for 60 seconds. After rinsing with water and air drying, the corresponding intermediate adhesive (Single Bond Universal Adhesive, 3M ESPE) was applied to the surfaces using a micro-brush and light cured for 10 seconds. Cement the S-FPDs with adhesive resin cement (RelyX™ Ultimate, 3M ESPE) (Figure 4).

(5) Finishing the restoration

Remove the excessive cementation. Check the occlusion. If one tooth included in the splint restoration is in a traumatic occlusion, the periodontal tissue of the remaining teeth may also be injured. So the S-FPDs restoration should not interfere with occlusion. Make sure there was no contact on the pontic part while protrusion as well as lateral excursions. There should be no contact on the adjacent teeth which were splinted during eccentric movement as well. For the maximum intercuspal position, the pontic part was adjusted less contact than adjacent natural teeth (about 30 *μ*m difference) in order to reduce the shear force applied to the restoration. Refine the surface of the S-FPDs after occlusal adjustment.

(6) Follow up

Recall the patient monthly for 3 months and then every 3 months to check the fitting and duration as well as cementation of the S-FPD restoration. Reinforce oral hygiene instruction and provide prophylaxis. Give X-ray examination at 6 months recall (Figure 5).

## 3. Discussion

After 6 months, this patient had acceptable oral hygiene and good control of periodontitis with no tooth mobility and further gingival recession (Figures 6(a) and 6(b)). On the basis of literature [17], lamina dura is a radiographic landmark viewed largely on periapical radiographs. The terminology lamina dura (or alveolus) is applied to the thin layer of dense cortical bone, which lines the roots of sound teeth. Presence of lamina dura is an indication of the health of the teeth. The periapical radiograph at 6 months recall (Figure 5) showed defined lamina dura at the crest of the bone around the adjacent natural incisors, which reminded bone regeneration.

This S-FPDs workflow is straightforward, convenient, and accurate. Due to the improved accuracy of the digital impression,^10^ the prosthesis is in good position when sitting. In addition, this S-FPDs is artistic and in favor of promoting periodontal health. Polished smooth surfaces help to control plaque and are well adapted to the arch curve and lingual profile of teeth, which improve patient's comfort. The splinting part of the restoration was designed with a minimal thickness of 1 mm. According to manufacture recommendations from other flexible PMMA brands, the minimal thickness could range from 0.6 mm (PMMA Disc, BEGO) to 0.8 mm (Telio CAD, Ivoclar). So further investigation might be needed to find a proper design not only ensure enough intensity but also improve the comfort of patients.

This technique did not need tooth preparation, so preserve as much enamel as possible. Bonding on enamel has been proved to be reliable. Together with the airborne-particle abrasion, supra gingival margins design, and careful adjustment on centric and eccentric occlusion, [18] the restoration has not shown breaking or loosening during 6 months and shown good function at 12 months recall (Figure 7).

PMMA material, whose physical properties have proven to be adequate for dental applications, was used in this case. The material is very popular for its ease of handling and manipulation, lack of toxicity, proper strength, and reasonable cost [19]. Moreover, the color, optical characteristics, and dimensional properties of PMMA remain stable under normal intraoral conditions. Under the demand for nonmetallic restorations from both clinicians and patients has encouraged researchers to seek alternative materials. PMMA blocks are fabricated at increased pressures and under strictly controlled thermal conditions [20]. It has decreased porosity, increased polymerization, a diminished residual monomer content, and is commonly used for prosthetic dental applications, including the fabrication of artificial teeth, denture bases, dentures, obturators, orthodontic retainers, temporary or provisional crowns, and for the repair of dental prostheses. It also has additional use for occlusal splints, printed or milled casts, and dies for treatment planning according to literature [21].

The flexible multilayered PMMA block has acceptable flexural strength, which is over 120 MPa according to the data from manufacture, and demonstrates significant superiority in surface wettability, surface roughness, and surface hardness [22]. Surface roughness has been described as “little indentations or irregularities that characterizes a surface and has its influence on wetting, quality of adhesion, and brightness of that surface.” [23] Less surface roughness can be more tolerable to discoloration and increase patient comfort. As mentioned in the literature [24], the Ra of CAD/CAM PMMA is around 0.2 *μ*m, which is below the threshold for plaque accumulation. Surface hardness is defined as “the ability of a material's surface to resist permanent penetration or indentation. “ [25] It has been reported that there is a correlation between surface hardness and material mechanical properties [26]. The prefabricated PMMA blocks are more resistant to fracture and have less chance of plaque, microorganism, and pigment retention, in turn increase the longevity of restoration. After 12 months restoration, the lingual surface of RB-S-FDP showed neither plaque nor pigment accumulation (Figure 7(b)), but a small amount of calculus was found in the interdental space due to inefficient oral hygiene (Figure 7(a)).

As a medium-term provisional restoration method, the adhesion is important for its durability. Adhesion has two aspects, and not only the tooth surface but also the conditioning of the restorative material is crucial for adequate bonding of the resin cement. For the RB-S-FDP, because the lower margin was designed within cingulum, the tooth surface for bonding was enamel, which has a nice result with etching-and-rinse bonding systems.

According to the literature [27], no adhesion of the cements was observed on unconditioned polymeric CAD/CAM crowns. One of the most common methods of conditioning polymeric materials is the use of airborne-particle abrasion, which in principle cleans the surface and at the same time increases the surface area. Airborne-particle abrasion before cementation of polymeric CAD/CAM material minimally improved the tensile strength.

Another common method of conditioning is the use of MMA-based liquid. But literature [28] reported that single use for MMA-based liquid, such as SR Connect, cannot attain adequate retentive strength. This could be explained by the high density of the PMMA block with a high degree of conversion. The highly cross-linked PMMA surface probably impeded the penetration of the MMA-based liquid and prevented the secondary interpenetrating polymer network bonding.

The combined application of both conditioning methods, which is airborne-particle abrasion and SR Connect, used in this case is recommended. The use of airborne-particle abrasion surface treatment most likely removed the outer dense layer on the PMMA restoration, so facilitating the penetration of the MMA-based liquid deeper into the surface, which enhanced the softening of the PMMA with the monomer.

The patient is satisfied with the aesthetic outcome of multilayered PMMA material. However, for higher aesthetic demand, cutback and staining would be needed. Long-term stability of this S-FPDs restoration and the effectiveness of this technique should be further evaluated with prospective clinical trial.

## Figures and Tables

**Figure 1:** Clinical situation after initial periodontal therapy.

**Figure 2:** Intraoral scan of both dentitions.

**Figure 3:** CAD-CAM procedure.

**Figure 4:** Immediate after cementation.

**Figure 5:** Periapical film of 6 months recall.

**Figure 6:** Clinical situation of 6 months recall.

**Figure 7:** Clinical situation of 12 months recall.

## Data Availability

The data that support the findings of this study are available from the corresponding author upon reasonable request.

## References

[1] Michaud D. S., Fu Z., Shi J., Chung M. (2017). Periodontal disease, tooth loss, and cancer risk. *Epidemiologic Reviews*.

[2] American Academy of P (2001). *Glossary of Periodontal Terms*.

[3] Tarnow D. P., Fletcher P. (1986). Splinting of periodontally involved teeth: indications and contraindications. *The New York State Dental Journal*.

[4] Li A., Chen L., Thomas R. Z. (2021). Periodontal breakdown inter-tooth relationships in estimating periodontitis- related tooth loss. *Journal of Dentistry*.

[5] McArthur D. R. (1985). Determination of approximate size of maxillary anterior denture teeth when mandibular anterior teeth are present. Part III: Relationship of maxillary to mandibular central incisor widths. *The Journal of Prosthetic Dentistry*.

[6] Liu X., Zhang Y., Zhou Z., Ma S. (2016). Retrospective study of combined splinting restorations in the aesthetic zone of periodontal patients. *British Dental Journal*.

[7] Minami H., Minesaki Y., Suzuki S., Tanaka T. (2012). Twelve-year results of a direct-bonded partial prosthesis in a patient with advanced periodontitis: a clinical report. *The Journal of Prosthetic Dentistry*.

[8] Wyatt C. C. (2007). Resin-bonded fixed partial dentures: what's new?. *Journal of the Canadian Dental Association*.

[9] Schlenz M. A., Schmidt A., Wöstmann B., Ruf S., Klaus K. (2019). In vitro comparison of analog versus digital impressions of the periodontally compromised dentition focused on interdental areas. *International Journal of Computerized Dentistry*.

[10] Schlenz M. A., Schubert V., Schmidt A., Wöstmann B., Ruf S., Klaus K. (2020). Digital versus conventional impression taking focusing on interdental areas: a clinical trial. *International Journal of Environmental Research and Public Health*.

[11] Kihara H., Hatakeyama W., Komine F. (2020). Accuracy and practicality of intraoral scanner in dentistry: a literature review. *Journal of Prosthodontic Research*.

[12] Mangano F., Gandolfi A., Luongo G., Logozzo S. (2017). Intraoral scanners in dentistry: a review of the current literature. *BMC Oral Health*.

[13] Deferm J. T., Schreurs R., Baan F. (2018). Validation of 3D documentation of palatal soft tissue shape, color, and irregularity with intraoral scanning. *Clinical Oral Investigations*.

[14] Rojo E., Stroppa G., Sanz-Martin I., Gonzalez-Martín O., Alemany A. S., Nart J. (2018). Soft tissue volume gain around dental implants using autogenous subepithelial connective tissue grafts harvested from the lateral palate or tuberosity area. A randomized controlled clinical study. *Journal of Clinical Periodontology*.

[15] Lee J. S., Jeon Y. S., Strauss F. J., Jung H. I., Gruber R. (2020). Digital scanning is more accurate than using a periodontal probe to measure the keratinized tissue width. *Scientific Reports*.

[16] Zhang C., Liu Q., Yang J., Hou J. (2021). A digital technique for splinting periodontally compromised mobile teeth in the mandibular anterior region. *The Journal of Prosthetic Dentistry*.

[17] Prakash N., Karjodkar F. R., Sansare K., Sonawane H. V., Bansal N., Arwade R. (2015). Visibility of lamina dura and periodontal space on periapical radiographs and its comparison with cone beam computed tomography. *Contemporary clinical dentistry*.

[18] Balasubramaniam G. R. (2017). Predictability of resin bonded bridges - a systematic review. *British Dental Journal*.

[19] Babu M. R., Rao C. S., Ahmed S. T., Bharat J. S. V., Rao N. V., Vinod V. (2014). A comparative evaluation of the dimensional accuracy of heat polymerised PMMA denture base cured by different curing cycles and clamped by R S technique and conventional method - an in-vitro study. *Journal of International Oral Health: JIOH*.

[20] Lauvahutanon S., Takahashi H., Shiozawa M., Iwasaki N., Asakawa Y., Oki M. (2014). Mechanical properties of composite resin blocks for CAD/CAM. *Dental Materials Journal*.

[21] Zafar M. S. (2020). Prosthodontic applications of polymethyl methacrylate (PMMA): an update. *Polymers (Basel)*.

[22] Al-Dwairi Z. N., Tahboub K. Y., Baba N. Z., Goodacre C. J., Özcan M. (2019). A comparison of the surface properties of CAD/CAM and conventional polymethylmethacrylate (PMMA). *Journal of Prosthodontics*.

[23] Cortés-Sandoval G., Martínez-Castañón G. A., Patiño-Marín N., Martínez-Rodríguez P. R., Loyola-Rodríguez J. P. (2015). Surface roughness and hardness evaluation of some base metal alloys and denture base acrylics used for oral rehabilitation. *Materials Letters*.

[24] Alp G., Johnston W. M., Yilmaz B. (2019). Optical properties and surface roughness of prepolymerized poly(methyl methacrylate) denture base materials. *The Journal of Prosthetic Dentistry*.

[25] Abdulwahhab S. S. (2013). High-impact strength acrylic denture base material processed by autoclave. *Journal of Prosthodontic Research*.

[26] Lee H. H., Lee C. J., Asaoka K. (2012). Correlation in the mechanical properties of acrylic denture base resins. *Dental Materials Journal*.

[27] Stawarczyk B., Basler T., Ender A., Roos M., Ozcan M., Hämmerle C. (2012). Effect of surface conditioning with airborne-particle abrasion on the tensile strength of polymeric CAD/CAM crowns luted with self-adhesive and conventional resin cements. *The Journal of Prosthetic Dentistry*.

[28] Pitta J., Bijelic-Donova J., Burkhardt F., Fehmer V., Närhi T., Sailer I. (2020). Temporary implant-supported single crowns using titanium base abutments: an in vitro study on bonding stability and pull-out forces. *The International Journal of Prosthodontics*.

